# Integrin-linked kinase affects the sensitivity of esophageal squamous cell carcinoma cells to chemotherapy with cisplatin via the Wnt/beta-catenin signaling pathway

**DOI:** 10.1080/21655979.2022.2076497

**Published:** 2022-05-19

**Authors:** Ting Xu, Xiao-Li Ma, Yu Wei, Lei-Yu Cao, Yan Gao, Juan Liu, Li Zhang

**Affiliations:** a Department of Internal Medicine 1, the First Affiliated Hospital of Xinjiang Medical University, Urumqi, Xinjiang Uygur Autonomous Region, China; b Department of Internal Medicine 4, the First Affiliated Hospital of Xinjiang Medical University, Urumqi, Xinjiang Uygur Autonomous Region, China

## Abstract

Recent studies have shown that the expression of integrin-linked kinase (ILK) was related to the occurrence, development, and malignant progression of esophageal squamous cell carcinoma (ESCC). However, research on the relationship between ILK and the chemosensitivity of ESCC has to date not been reported. The present study found that ILK was highly expressed in ESCC cell lines, and the overexpression of ILK in ESCC cells reduced the incidence of cell apoptosis and alleviated the cytotoxicity on cells induced by cisplatin (CDDP). Inversely, ILK knockdown increased CDDP-induced apoptosis and had an inhibitive effect on the malignant phenotype of ESCC, including cell proliferation, invasion, and migration. In addition, ILK knockdown in ESCC cells inhibited the expression of beta (β)-catenin and activated the wingless/integrated (Wnt) signaling pathway. Furthermore, cellular MYC (c-MYC) and Cylin D1 were the target genes of the Wnt signaling pathway. Rescue experiments showed that the overexpression of β-catenin reversed a tumor’s inhibition and apoptosis abilities induced by ILK knockdown. In conclusion, ILK potentially reduced the CDDP sensitivity of ESCC cells by influencing the activity of the Wnt/β-catenin signaling pathway.

## Highlights

- Integrin-linked kinase (ILK) was highly expressed in esophageal squamous cell carcinoma (ESCC) cell lines.
- The overexpression of ILK reduced the chemosensitivity of ESCC cells to cisplatin (CDDP).
- The downregulation of ILK increased the sensitivity of ESCC cells to CDDP chemotherapy.
- ILK-mediated sensitivity to CDDP chemotherapy is involved in the wingless/integrated/beta-catenin pathway.

## Introduction

In China and elsewhere in the world, esophageal carcinoma (EC) is one of the most malignant tumors. According to survey data collected by the International Agency for Research on Cancer, in 2020, approximately 604,100 new cases of EC were recorded worldwide, accounting for 3.1% of all cancers [1]. According to histological data, EC can be divided into two types, i.e., esophageal squamous cell carcinoma (ESCC) and esophageal adenocarcinoma. In Europe and the United States, the primary histological type of EC is adenocarcinoma, while in China, the proportion of ESCCs is higher than 90% [2,3]. Presently, the treatment of EC is primarily surgery, followed by radiotherapy and chemotherapy.

Although surgery, chemotherapy, and radiation therapy have improved over the past decades, the clinical application of current medical interventions remains unsatisfactory [4]. As the most widely used chemotherapeutic drugs, current cisplatin (CDDP)-based chemotherapy regimens represent the preferred clinical treatment approach for advanced ESCC. CDDP mainly acts on the deoxyribonucleic acid (DNA) of cells and can cause DNA damage and induce cell apoptosis. However, during the course of CDDP-based chemotherapy, the occurrence of chemotherapy drug-resistance reduces the therapeutic effect and is the main reason for the poor prognosis and low five-year survival rate among ESCC patients, thus introducing challenges to anti-cancer chemotherapy [5,6]. Accordingly, understanding the molecular mechanism of chemotherapy resistance in ESCCs, exploring new targets for chemotherapy resistance, and promoting the development of new therapeutic agents has important clinical significance for improving curative effects and survival rates.

Integrin-linked kinase (ILK) is a widely expressed serine/threonine-specific protein kinase that is located in focal adhesions and plays a critical role as a multifunctional effector of growth factor signaling and cell-matrix interactions [7,8]. According to reports, ILK is overexpressed in colorectal cancer, bladder cancer, and many other tumor tissue types and is associated with TNM (‘tumor,’ ‘nodes,’ and ‘metastasis’) stage, lymph node metastasis, and differentiation, thus indicating ILK as a potential anti-cancer therapeutic target [9–12].

ILK is also involved in cell proliferation, differentiation, invasion, and metastasis through a variety of signaling pathways, including the classic wingless/integrated signaling (Wnt/beta (β)-catenin) pathway. The ability of ILK to activate the Wnt/β-catenin signaling pathway by increasing the expression level of β-catenin, the key protein of the Wnt/β-catenin pathway, has been reported, thereby participated in the malignant behavior of a variety of tumors [13,14].

In addition, the involvement of ILK has also been reported in the regulation of chemotherapeutic sensitivity. For example, Duxbury et al. [15] reported that the overexpression of ILK in pancreatic cancer cells could enhance cell resistance to gemcitabine, while ILK knockdown could increase caspase-3-mediated apoptosis and increase cell sensitivity to gemcitabine. Yau et al. [16] found that the use of ILK inhibitor QLT0254, combined with gemcitabine, could increase the drug sensitivity of gemcitabine in a mouse model of orthotopic pancreatic tumors. However, the function of ILK as it concerns the chemosensitivity of ESCC has to date not been fully elucidated.

Based on the outcomes of several studies, the Wnt/β-catenin signaling pathway also plays an important role in the CDDP resistance of various tumors. It has been reported that β-catenin gene-silencing led to the inhibition of Wnt signaling pathway activity, which reduced CDDP resistance in head and neck squamous cell carcinoma and epithelial ovarian carcinomas cells [17,18]. However, its role in the sensitivity of CDDP chemotherapy in ESCCs has not been fully elucidated.

The current research team confirmed that ILK was highly expressed in the peripheral blood of ESCC patients and that this was related to the efficacy of radiotherapy and chemotherapy [19]. Additionally, the in vitro experiments of these studies have also demonstrated that silencing ILK expression could inhibit the proliferation, invasion, and metastases of ESCC cells [19]. Therefore, the purpose of the present study was to further explore the role of ILK in chemotherapy sensitivity for ESCCs. The study results suggested that the overexpression or knockdown of ILK could significantly affect the chemosensitivity of ESCC cells to CDDP and that this effect may be mediated by affecting the expression level of β-catenin, which is the key protein for activation of the Wnt/β-catenin signaling pathway.

## Materials and methods

### Cell culture

Five human ESCC cell lines (EC109, KYSE150, TE-1, KYSE30, and EC9706) and one esophageal epithelial cell line (SHEE) were purchased from the Cell Bank of the Chinese Academy of Science (Shanghai, China). All of the cells were cultured in Dulbecco’s Modified Eagle Medium (DMEM) (Invitrogen, Carlsbad, CA, USA) containing 10% fetal bovine serum (FBS) (Gibco, Rockville, MD, USA), 100 IU/mL streptomycin, and 100 IU/mL penicillin (Sigma, St. Louis, MO, USA) in a humidified atmosphere (37°C, 5% carbon dioxide).

### Quantitative real-time polymerase chain reaction

TRIzol (Invitrogen, Carlsbad, CA, USA) was used to extract total ribonucleic acid (RNA) from ESCC cells. A Prime Script RT reagent kit (Takara Bio Inc, Otsu, Japan) was used to synthesize the first-strand complementary DNA. Real-time polymerase chain reactions (RT-PCR) were performed using an Applied Biosystems® 7500 Real-time PCR system (Thermo Fisher Scientific, Foster, CA, USA). The included primers were as follows ILK, forward: 5′-TTAGCATGGCTGATGTCAAGTTC-3’, reverse: 5′-TCTGCTGAGCGTCTGTTTGTG-3′; glyceraldehyde 3-phosphate dehydrogenase (GAPDH), forward: 5′-ATCCCATCACCATCTTCCAGG-3′, and reverse: 5′-GATGACCCTTTTGGCTCCC-3′. The relative gene expression was normalized to GAPDH and quantified by the 2^− delta–delta Ct^ (2^−ΔΔCt^) method.

### Western blot analysis

The proteins were separated by 10% sodium dodecyl sulfate-polyacrylamide gel electrophoresis (40 μg each) and then transferred to a polyvinylidene fluoride membrane (Millipore, Boston, MA, USA). The membrane was then sealed with 5% skim milk in Tris-buffered saline containing 0.1% (v/v) Tween 20 at pH 7.6 for 1 h and incubated overnight with a primary antibody at 4°C (primary antibody: ILK [1:3,000, Abcam, Cambridge, MA, USA], β-catenin [1:3,000, Abcam, Cambridge, MA, USA], c-MYC, Cylin D1 [1:100, Santa Cruz Biotechnology, CA, USA], and GAPDH [1:500, Affinity Biosciences, OH, USA]). The membrane was then rinsed and incubated with horseradish peroxidase labeled goat anti-rabbit immunoglobulin G (IgG) secondary antibody(1:1000, Santa Cruz Biotechnology, CA, USA) or alkaline phosphatase labeled goat anti-rabbit immunoglobulin G (IgG) secondary antibody(1:1000, Biorab, Beijing, China). The bands were detected by ECL Western blotting reagent (Amersham, Piscataway, NJ, USA) or AP Western Detection Kit (Thermo Fisher Scientific, USA). Quantity One (Version 4.6.2) imaging software (Bio-Rad, Hercules, CA, USA) was used for computer analysis of the band pixel intensity.

### Lentivirus vectors and transfection

Three pairs of short hairpin RNA-targeting ILK lentivirus vectors and overexpression vectors were specifically synthesized by Jikai Technologies (Shanghai, China). Activated β-catenin (s33y) mutants were previously described in detail [20]. Next, TE-1 and KYSE150 cells were transfected with vectors, respectively. Knockdown or overexpression efficiency was measured at 48 h post-transfection by Western blotting and RT-PCR.

### In vitro chemosensitivity assay

The adopted cell density was 1 × 10^4^ cells per well. The cells were inoculated in 96-well plates overnight and treated with a corresponding concentration of CDDP (Sigma-Aldrich, Saint Louis, USA) in a specific environment at 37°C; a time limit of 24 h was adopted. Next, cell counting kit-8 (CCK-8) (10 μL) (Beyotime Biotechnology, Shanghai, China) was added to each well individually and cultured at 37°C in a specific environment for 1 h. The optical density (OD) was accurately measured at 450 nm by an enzyme-linked immunosorbent assay microplate reader (Bio-Rad). Cell viability = (the OD value of the experimental group – the OD value of the blank group)/(the OD value of the control group – the OD value of the blank group) × 100%. Three different independent experiments were carried out in turn. The half-maximum inhibitory concentration (IC50) was calculated using GraphPad Prism 5.0 to study and evaluate the ready state and drug resistance of cells to CDDP.

### Colony formation assay

Esophageal squamous cell carcinoma cells were inoculated into 6-well plates at a density of 1.5 × 10^3^ cells per well and treated with CDDP at the corresponding concentration. After 10–14 days of culture, the cells were immobilized with ethanol for 30 min and then stained with 0.1% crystal violet for 15 min. Clones with ≥50 cells were counted. All assays were independently performed in triplicate.

### Wound-healing assay

The transfected ESCC cells that had reached the logarithmic growth stage (CDDP-treated/not-CDDP-treated) were digested by trypsin, centrifuged, and suspended in a DMEM (10% FBS) medium. The cell concentration was adjusted to 3 × 10^5^/mL, and a 100- μL cell suspension was added to the 6-well cell-culture plate and cultured until the cell density was higher than 90%. When this cell density was achieved, the supernatant culture medium was removed and a new culture medium was added. Scratches were then formed on the bottom of the cell culture plate using a scratch meter. The cells were washed 2–3 times in a DMEM medium and photographed after adding 0.5% FBS. The culture process was continued, observed, and photographed at 0, 24, and 48 h, respectively. At least four wound locations or areas had to be photographed in each plate to facilitate measurement migration.

### Transwell migration and invasion assays

In the migration and invasion experiments, the ESCC cells in each group were treated with CDDP at the corresponding concentration at 37°C for 24 h, and the treated cells were suspended in a serum-free medium at a density of 1 × 10^5^ cells per well and seeded at the upper transwell chamber insert(Corning Costar, NY, USA). For the invasion assay, the treated cells were inoculated into the upper chamber, pre-coated with 20 μg Matrigel (BD Bioscience, CA, USA) at a density of 1 × 10^5^ cells per well. For both tests, 500 μl of DMEM containing 20% FBS was added to the lower lumen. After 24 h, the remaining cells in the front of the upper chamber were gently wiped clean using cotton swabs, and the cells in the back of the chamber were fixed, stained with 0.1% crystal violet for 30 min, and calculated under a microscope (Olympus, Tokyo, Japan) by counting five separate visual fields.

### Cell apoptosis analysis

Apoptosis in the ESCC cells treated with or without CDDP was assessed using an Annexin V-FITC/propidium iodide (PI) kit (Beyotime, Shanghai, China). Briefly, the cells were digested, cleaned, and centrifuged with cold phosphate-buffered saline (PBS). Annexin V-FITC and PI were used for staining at room temperature (30 min). Then, the cells were detected by flow cytometry (Becon Dickinson Facsalibur, USA). The FlowJo (Version 10.0.7, Ashland, OR, USA) software program was used to quantify the data.

### Tumor xenograft models

The living conditions of mice were specific pathogen-free grade. The environmental temperature was 26°C–28°C, and the light and dark cycles were 12 and 12 h, respectively. Mice were fed sterile food and water, which was sterilized by high-pressure steam. Thirty four-week-old female BALB/c nude mice (Shanghai Experimental Animal Center, Chinese Academy of Sciences, Shanghai, China) were randomly divided into six groups (n = 3). Then, the oe-NC(lentivirus overexpressing negtive control vector), oe-ILK(lentivirus overexpressing ILK), sh-ILK (lentivirus expression shRNA against ILK), and sh-NC (lentivirus expression shRNA against ILK negative control) of TE-1 cells were collected, respectively, and a cell suspension containing 6 × 10^6^ cells/mL was prepared. Each mouse was subcutaneously injected with 100 µL of the abovementioned cell suspension into the right axilla. When the maximum tumor diameter reached 5 mm, CDDP (2 mg/kg, twice a week) or an equivalent PBS was injected intraperitoneally over three weeks. The tumor volume (mm^3^) = (length × width^2^)/2. On day 30, the mice were euthanized by cervical dislocation. Concurrently, the transplanted tumor tissue was resected and weighed. All procedures were approved by the Institutional Animal Care and Use Committee of Xinjiang Medical University (IACUC-20200715-01) and conformed to the National Institutes of Health’s Guide for the Care and Use of Laboratory Animals.

### Immunohistochemistry staining

The tissue wax blocks were sectioned on a paraffin slicer with a thickness of 4 μm. After dewaxing, 3% hydrogen peroxide solution was added and treated at room temperature for 10 min, followed by treatment with 5% BSA(Ameresco, OH, USA) for 20 min. Drop Ki67 (1:300, Abcam, Cambridge, MA, USA) primary antibody working solution overnight at 4°C. Then the pre-diluted biotin-labeled secondary antibody(1:1000, Biorab, Beijing, China) was added and treated at 37°C for 30 min, then incubated with HRP-labeled avidin(Bersee, Beijing, China) incubate at 37°C for 30 min. After cleaning with PBS solution, DAB(Beyotime Biotechnology, Shanghai, China) solution was prepared with 80 μL fresh for each slices, and washed with distilled water. Then, the slices were stained with hematoxylin for 25s, and washed with running water for 3 min. The slices were dehydrated, sealed with neutral gum, dried in a ventilated kitchen, and placed under a microscope(Olympus, Tokyo, Japan) for observation and image collection and analysis.

### Tunel assay

After dewaxed, paraffin slices were immersed in a PBS staining tank containing 4% paraformaldehyde and placed at 4°C for 25 min for cell fixation. Add 100 μL diluted Proteinase K solution to each slice, and incubate at room temperature for 5 min for permeability treatment. Add 50 μL TUNEL (Vazyme, Nanjing, China) and incubate for 1 h. The samples were restained with 2 μg/mL DAPI solution freshly prepared with PBS in the dark for 5 min. Results were observed and collected under a fluorescence microscope(Olympus, Tokyo, Japan).

### Statistical analysis

Data analysis was performed using SPSS 21.0 (IBM, Chicago, IL, USA). Data are presented as mean ± standard deviation. A paired t test was used to compare two sets of paired data. Comparison of two sets of unpaired data was performed by unpaired t test. The statistical analysis between each group was carefully analyzed using an independent sample t-test and one-way analysis of variance. A value of P < 0.05 was considered to indicate statistical significance.

## Results

### The expression level of integrin-linked kinase in esophageal squamous cell carcinoma cells

We examined the expression of ILK in five ESCC cell lines (KYSE150, EC9706, KYSE30, TE-1, and EC109) and one esophageal epithelial cell line (SHEE). The RT-PCR results showed that the expression of ILK was significantly higher in all five ESCC cell lines compared with the SHEE cells (Figure 1a). The Western bolt results showed that ILK expression was significantly higher in KYSE150, EC9706, TE-1, and EC109 cells compared with the SHEE cells (Figure 1b).

**Figure 1.** The expression level of ILK in ESCC cells. (a) ILK detected by RT-PCR in five ESCC cell lines and one esophageal epithelial cell line (SHEE). (b)WB analysis of ILK expression in ESCC cell lines and SHEE.*p < 0.05,**p < 0.01.

### The expression of integrin-linked kinase is associated with the chemosensitivity of esophageal squamous cell carcinoma cells to cisplatin

To study the effect of downregulation and the overexpression of ILK on the behaviors of ESCC cells simultaneously, TE-1 and KYSE150 cells with moderate ILK expression were used for the following experiments.

To explore the relationship between ILK expression and the chemosensitivity of CDDP, the CCK-8 assay was used to detect the effect of CDDP on the proliferation of TE-1 and KYSE150 cells in the overexpressed ILK group (oe-ILK) and ILK knockdown group (sh-ILK), as well as corresponding control groups (oe-NC and sh-NC). The IC50-to-CDDP of oe-ILK-transfected TE-1 and KYSE150 cells was significantly higher compared with the negative control (oe-NC) (Figure 2(e,g)), while the IC50-to-CDDP of sh-ILK transfected TE-1 and KYSE150 cells showed a significant decrease compared with the negative control group (sh-NC) (Figure 2(f,h)). These results suggested that the overexpression of ILK could increase the IC50 of TE-1 and KYSE150 to CDDP, while ILK knockdown decreased the IC50 of TE-1 and KYSE150 to CDDP.

**Figure 2.** ILK affects ESCC sensitivity to DDP. (a-d) Relative expression of ILK was assayed in KYSE150 and TE-1 cells infected with oe-ILK(overexpression of ILK) or sh-ILK (konckdown of ILK) by WB. (e-f) The IC50 of TE-1 to CDDP after transfection with oe-ILK and sh-ILK. (g-h) The IC50 of KYSE150 to CDDP after transfection with oe-ILK and sh-ILK. *p < 0.05, **p < 0.01.

### The effects of integrin-linked kinase on the proliferation of esophageal squamous cell carcinoma cells via treatment with cisplatin

The proliferation of transfected cells treated with CDDP was detected using a clonal formation assay. The results showed that CDDP could significantly inhibit the cloning ability of TE-1 and KYSE150 cells (Figure 3(a–d)). The overexpression of ILK reduced the inhibiting effect of CDDP on the cloning ability of ESCC cells (Figure 3(a,c)), while the downregulation of ILK expression further aggravated the inhibiting effect of CDDP on cell colony formation (Figure 3(b,d)).

**Figure 3.** Effects of ILK on the proliferation of ESCC cells toward CDDP. (a-b) Proliferative capacity of TE-1 exposed to DDP after transfection with oe-ILK and sh-ILK was analyzed by colony formation assay. (c-d) Proliferative capacity of KYSE150 exposed to DDP after transfection with oe-ILK and sh-ILK was analyzed by colony formation assay.^*#^*p* < 0.05 and ^**##^p < 0.01.

### The effects of integrin-linked kinase expression on the apoptosis of esophageal squamous cell carcinoma cells via treatment with cisplatin

To examine the effect of ILK on the apoptosis of ESCC cells, flow cytometry was used to detect the CDDP-induced apoptosis of TE-1 and KYSE150 cells in the oe-ILK and sh-ILK groups, as well as the oe-NC and sh-NC groups. Transfection with oe-ILK significantly reduced the percentage of apoptotic cells treated with CDDP compared with the negative control (Figure 4(a,c)). Transfection with sh-ILK significantly increased the percentage of apoptosis after CDDP treatment (Figure 4(b,d)). These results indicated that the up-regulation of ILK expression could alleviate the sensitivity of CDDP chemotherapy and reduce the apoptosis caused by CDDP treatment. The downregulation of ILK expression could enhance the chemotherapy response to CDDP and increase the apoptosis of ESCC cells.

**Figure 4.** Effection of ILK on apoptosis of ESCC cells toward to CDDP. (a-b) Cell apoptosis of TE-1 induced by CDDP after transfection with oe-ILK and sh-ILK was analyzed with flow cytometry. (c-d) Cell apoptosis of KYSE150 induced by CDDP after transfection with oe-ILK and sh-ILK was analyzed by flow cytometry. *^#^p* < 0.05 and ^**##^p < 0.01.

### The effects of integrin-linked kinase expression on the migration and invasion of esophageal squamous cell carcinoma cells via treatment with cisplatin

Wound-healing (Figure 5) and Transwell experiments (Figure 6) were performed to study the effects of ILK overexpression and knockdown on the migration and invasion metastasis of ESCC cells (TE-1 and KYSE150) under treatment with CDDP. The results showed that the overexpression of ILK alleviated the inhibitory effect of CDDP on ESCC cell migration, while interference with ILK expression further aggravated the inhibitory effect of CDDP on ESCC cell migration and invasion.

**Figure 5.** Effects of ILK on ESCC cell migration to CDDP. (a-b) Effect of ILK on cell migration toward CDDP was assessed by wound healing assays in TE-1. (c-d) Effect of ILK on cell migration toward CDDP was assessed by wound healing assays in KYSE150. *^#^p* < 0.05 and ^**##^p < 0.01.

**Figure 6.** Effects of ILK on ESCC cell migration and invasion to CDDP. (a-b) Effect of ILK on cell migration toward CDDP was assessed by Transwell assays without Matrigel in TE-1. (c-d) Effect of ILK on cell migration toward CDDP was assessed by Transwell assays without Matrigel in KYSE150. (e-f) Effect of ILK on cell invasion toward CDDP was assessed by Transwell assays with Matrigel in TE-1. (g-h) Effect of ILK on cell invasion toward CDDP was assessed by Transwell assays with Matrigel in KYSE150. ^*#^p < 0.05 and **p < 0.01.

### The knockdown of integrin-linked kinase promotes the sensitivity of esophageal squamous cell carcinoma cells to cisplatin by affecting the expression level of beta-catenin

To investigate the role of ILK on the above processes, TE-1 cell line was selected to perform the knockdown and rescue experiment, because of its relatively higher ILK expression than that of KYSE150 cells. Western blot analysis showed that knockdown of ILK downregulated the expression of β-catenin, c-MYC, and Cylin D1, as well as the expression of drug-resistance-related protein MDR1 (Figure 7a). To explore the potential mechanism of ILK in the chemotherapeutic sensitivity of ESCC cells to CDDP, a rescue experiment was conducted, ILK-Knockdown cells co-transfected with β-catenin. The results showed that the overexpression of β-catenin could alleviate the inhibition of proliferation (Figure 7b), migration and invasion (Figure 7(d–f)), as well as could inhibit the apoptosis of TE-1 cells (Figure 7c) caused by ILK knockdown via CDDP treatment. These results suggested that ILK may affect the chemotherapy sensitivity of ESCC cells through the expression level of β-catenin, which is a key protein of the Wnt/β-catenin signaling pathway.

**Figure 7.** Knockdown of ILK promotes the sensitivity of ESCC cells to CDDP through disturbing the expression of β-catenin. (a) The expression level of ILK, β-catenin, c-MYC, MRD1 Cylin D1, level was detected by WB in TE-1 cells after transfected with sh-ILK and sh-NC. (b) Effects of β-catenin overexpression on cell colony formation to CDDP after knockdown of ILK. (c) Effects of β-catenin overexpression on cell apoptosis to CDDP after knockdown of ILK. (d-e) Effects of β-catenin overexpression on cell migration to CDDP after knockdown of ILK by wound healing assays and Transwell assays (without Matrigel). (f) Effects of β-catenin overexpression on cell invasion to CDDP after knockdown of ILK by transwell assays (with Matrigel).^* #^p < 0.05 and **p < 0.01.

### The effects of ILK expression on the xenograft tumor formation by esophageal squamous cell carcinoma cancer cells in vivo toward cisplatin treatment

Additional TE-1 cells were selected as experimental cells in this part of the study, and the experiment was divided into PBS-sh-NC, PBS-oe-NC, CDDP + sh-NC, CDDP + oe-NC, CDDP + sh-ILK, and CDDP + oe-ILK groups. The cells in each group were cultured to the required number and thereafter subcutaneously inoculated to establish an internal transplanted tumor model in nude mice. CDDP or PBS was intraperitoneally injected to observe the effect of changes in ILK expression on the tumor formation in nude mice. The results showed that CDDP could significantly reduce the tumor weight and volume in the CDDP-oe-NC compared with the PBS–oe-NC groups; ILK overexpression also significantly restored the reduction of tumor weight and volume induced by CDDP compared with the CDDP + oe-NC group (Figure 8(a,c)), while ILK knockdown could further reduce the weight and volume of tumors after treatment with CDDP (Figure 8(b,d)). Moreover, immunohistochemistry and terminal deoxynucleotidyl transferase assay (TUNEL assay) were used to detect tumor growth and apoptosis. The results showed that, compared with the PBS treatment groups, the CDDP treatment could reduce the positive rate of Ki67 and enhance the level of apoptosis of cells in tumor tissues. The overexpression of ILK could alleviate the promotion of apoptosis and the proliferation inhibition induced by CDDP treatment to some extent (Figure 8(e,g)), while the interference of ILK could further enhance the inhibition caused by CDDP on cell proliferation and apoptosis promotion (Figure 8(f,h)). Based on the above results, the present study posits that ILK may also affect the sensitivity of ESCC cells to CDDP chemotherapy in vivo.

**Figure 8.** Effects of ILK expression on the xenograft tumor formation by ESCC cancer cells in vivo toward CDDP treatment. (a-b) The tumor volume of each group. (c-d)The tumor weight from the xenografts all mice were killed at the end of the experiment. (e) Cell apoptosis in each group was assessed by TUNEL (f) The expression of cell proliferation related protein Ki67 in each group was detected by Immunohistochemistry. ^*#^p < 0.05 and ^**##^p < 0.01.

## Discussion

The progression of ESCC involves multiple steps, from precancerous lesions to aggressive ESCC. Since there are no early symptoms or signs for recognizing ESCC, most patients with ESCC are diagnosed at an advanced stage, which contributes to a poor prognosis [21]. The most common treatment for advanced ESCC is CDDP-based chemotherapy; however, only 2%–50% of patients respond well to this approach. Unlike other types of tumors, targeted therapies for ESCC have not significantly progressed [22]. Therefore, exploring the genes associated with cancer development and chemotherapy resistance in ESCC may contribute to the diagnosis, prognosis, prediction, and development of new treatment strategies.

ILK was defined as a serine/threonine-protein kinase, which is a cellular effector of integrin receptors involved in a variety of biologically active signaling pathways, including integrin, growth factors and Wnt signaling pathways and it plays an important role in signal transduction mediated by extracellular matrix, regulates cell growth, differentiation, migration, apoptosis, adhesion, proliferation and cell cycle [23]. Moreover, due to its involvement in the regulation of a variety of cellular biological processes, it is associated with the occurrence, development, invasion, and metastases of malignant tumors, and, as such, affects the prognosis of these tumors [24]. It has been reported that ILK gene knockout can inhibit the invasion and metastasis of Renal Cell Carcinoma and breast cancer [11,25], and is also an attractive target for the treatment of ovarian cancer [26]. Previous experimental results derived by the authors’ team showed that the downregulation of ILK inhibited the proliferation and migration of ESCC cells, suggesting that ILK may play an important role in the progression of ESCC. In addition, the authors’ previous research also found that compared with a chemotherapy-resistant group, the expression of ILK in the peripheral blood of a radio-chemotherapy-sensitive group had been decreased, suggesting that ILK may have been involved in the regulation of radio-chemotherapy-sensitivity in ESCC patients [19].

Presently, the basic chemotherapy regimen for ESCC is CDDP-based adjuvant chemotherapy [27]. CDDP is a DNA damage alkylation agent that can induce cell apoptosis and death [28]. Although CDDP-based multidrug chemotherapy has greatly improved the prognosis of patients, the high incidence of CDDP resistance remains a major obstacle for chemotherapy in ESCC patients [29]. It is thus very important to establish the key molecules of CDDP chemotherapy resistance in ESCCs. In recent years, ILK has been reported as being involved in the drug-sensitivity of many types of tumors. For example, ILK could regulate the sensitivity of pancreatic cancer cells to gemcitabine [16], and the pharmacological inhibition of ILK in oncogene homolog (KRAS) mutant lung cancer cells could inhibit cell growth, migration, and epithelial mesenchymal transition, and increase sensitivity to CDDP chemotherapy [30]. These results suggested that ILK played an important role in the regulation of tumor sensitivity to chemotherapy.

In the present study, in vitro and in vivo experiments showed that the overexpression of ILK could increase the sensitivity of ESCC cells to CDDP, while knockdown of ILK could increase the sensitivity of ESCC cells to CDDP. In addition, the current study found that ILK knockdown inhibited the expression of MDR1 in ESCC cells. The products of the MDR1 gene are involved in the generation of multidrug resistance, and the chemotherapy resistance caused by MDR1 is one of the main causes of death among tumor patients [31–33]. Therefore, the results of the current study suggested that ILK may be an important regulator of drug resistance in cases of ESCC.

In this study, ILK knockdown significantly downregulated the expression levels of β-catenin, c-MYC, and Cylin D1 in ESCC cells. β-catenin has been established as a key protein of the classic Wnt signaling pathway(Wnt/β-catenin pathway), and c-MYC and Cylin D1 are downstream target proteins of β-catenin in the Wnt signaling pathway [17]. Existing studies have shown that the activity of the Wnt/β-catenin pathway plays an important role in the development of ESCC, while the inhibition of the Wnt/β-catenin pathway could also suppress the growth of ESCC cells [34,35]. The Wnt/β-catenin signaling pathway also plays an important role in the CDDP chemotherapy resistance of tumors, e.g., lung cancer and colon cancer [20, 36–38]. Alongside literature reviews, the current study proposes that the influence of ILK on the chemosensitivity of ESCC cells to CDDP is partly related to the Wnt/β-catenin signaling pathway. In this study, the authors designed rescue experiments to explore the potential mechanism of ILK in affecting the sensitivity of ESCC cells to CDDP chemotherapy by overexpressing β-catenin in ILK-knockdown ESCC cells, then the results of proliferation, migration, invasion, and apoptosis assays showed that the overexpression of β-catenin significantly reversed the ILK knockdown-induced sensitivity of ESCC cells to CDDP chemotherapy. Consequently, the authors propose that ILK could affect the chemosensitivity of ESCC cells to CDDP and that this effect may be mediated by affecting the expression of β-catenin, the key protein in the activation of the Wnt/β-catenin signaling pathway.

### Conclusion

This study found that the high expression of ILK in ESCC cell lines could reduce the chemosensitivity of ESCC cells to CDDP. In addition, ILK knockdown could inhibit the expression of β-catenin, c-MYC, and Cylin D1, as well as the expression of MRD1. Moreover, the overexpression of β-catenin in ILK knockdown cells could restore the inhibition of cells’ vitality induced by CDDP, indicating the possible inhibiting effect of ILK on the sensitivity to CDDP chemotherapy through the activation of the Wnt /β-catenin signaling pathway. These results may provide a new rational therapeutic target for ESCCs.

## Data Availability

We declared that materials described in the manuscript, including all relevant raw data, will be freely available to any scientist wishing to use them for non-commercial purposes, without breaching participant confidentiality. The datasets used and analysed during the current study available from the corresponding author.
